# Fear of COVID-19 infection and related factors in Japan: A comparison of college students, pregnant women, hospital nurses and the general public

**DOI:** 10.1371/journal.pone.0271176

**Published:** 2022-07-13

**Authors:** Kohei Koiwa, Koubun Wakashima, Michiko Ikuta, Keigo Asai, Gen Takagi

**Affiliations:** 1 Faculty of Education, Tohoku University, Sendai, Miyagi, Japan; 2 Graduate School of Health and Welfare, Kanagawa University of Human Services, Yokosuka, Kanagawa, Japan; 3 Graduate School of Education, Hokkaido University of Education, Kushiro, Hokkaido, Japan; 4 Faculty of Comprehensive Welfare, Tohoku Fukushi University, Sendai, Japan; Qazvin University of Medical Sciences, ISLAMIC REPUBLIC OF IRAN

## Abstract

The fear of COVID-19 has become a social problem during the pandemic. The present study compares the fear of COVID-19 among members of the general public, college students, pregnant women, and hospital nurses. It also examines various factors associated with the fear of COVID-19. In this study, we conducted a survey of the general public on fear of infection and related factors and compared from previous studies of college students, pregnant women, and hospital nurses. A crowdsourced survey was administered to 450 members of the general public, who were asked about their fear of COVID-19 infection. Data from college students, nurses, and pregnant women were recruited from a May-June 2020 survey on fear of COVID-19. An analysis of variance was used to compare the fear of infection among different attribution. The results showed that more pregnant women and fewer college students feared infection, as did equal numbers of hospital nurses and members of the general public. The multiple regression analysis revealed that college students and pregnant women associated the fear of infection with their key source of information, while hospital nurses associated the fear of infection with living with an older person. These results suggest that pregnant women have a significant fear of infection, which is further defined by the risk of serious illness in cases of infection. Although the fear of infection is relatively low among hospital nurses, they fear becoming a source of infection. These results reveal the groups in Japan that fear infection and the reasons for their concern. The present study may help to provide psychological support to counteract the fear of infection in vulnerable groups.

## Introduction

As of March 3, 2022, there have been 437,333,859 confirmed cases of COVID-19 and 5,960,972 deaths worldwide [1]. In Japan, 5,127,714 people have caught COVID-19 and 24,084 have died [2], while the virus continues to spread.

COVID-19, an unknown infectious disease, has had many psychological effects. A meta-analysis of mental health during the COVID-19 pandemic concluded that 31.4% of the general public experienced depressive symptoms, 31.9% experienced anxiety symptoms, and 41.1% experienced psychological distress [3]. Furthermore, in a review on insomnia, 24% of women and 27% of men reported sleep disorder symptoms [4].

Fear of infection with COVID-19 (hereinafter referred to as “fear of infection”) is thought to be the core psychological problem experienced during the COVID-19 pandemic [5]. An Iranian study has shown a significant association between the fear of infection among older people and various health issues, including insomnia, and mental health [6]. According to a Turkish study, the fear of infection has increased depression, anxiety, and stress among members of the general public [7]. In a Greek study, the public fear of infection was associated with anxiety disorders and post-traumatic stress disorder [8]. Alimoradi et al. [9], who synthesized these studies and conducted a meta-analysis, reported that fear of infection was moderately associated with mental health deterioration, including stress reactions and depressive symptoms. Furthermore, a review article on the relationship between fear of infection and attitudes toward work demonstrated that fear of infection was linked to future career uncertainty, job insecurity, decreased job satisfaction, and turnover intentions [10]. Thus, fear of infection has been reported to impact many psychosocial factors.

In psychological research on the fear of infection, a scale has been developed to measure the degree of anxiety and fear of COVID-19. This scale, known as the Fear of COVID-19 Scale (FCV-19S), has been validated for reliability and validity [11]. For FCV-19S, some studies assumed a single structure [12], while others suggested a two-factor structure [13]. These systematic reviews concluded that a one-factor structure was reasonable for FCV-19S [14]. Additionally, the FCV-19S has cleared the high factor loadings, normal distribution, ceiling and floor effect studies [12]. Therefore, it has been concluded to be an instrument of distinction that can adequately measure differences in fear among people of various ages, genders, and populations [14]. Furthermore, the FCV-19S has been translated into multiple languages in Bangladesh, the UK, Brazil, Italy, Pakistan, and France; it has also been used in an international study to compare the intensity of anxiety and fear of COVID-19 infection [15].

A Japanese version of the FCV-19S [16] has been developed and used to examine related factors. Based on this study, they have drawn the following two conclusions: (A) Following an analysis of the association between the fear of infection and factors such as smoking history, family structure, current health status, illnesses under treatment, and employment status, they found that only the most important information sources were significantly associated with fear of infection; (B) The psychosocial behaviors associated with COVID-19 have been grouped into three categories: “being careful in daily life” (continuing preventive behaviors against COVID-19), “stockpiling” (buying and stockpiling food and daily necessities), and “health monitoring” (observing one’s own health status). All of these behaviors are significantly associated with the fear of infection. The present study also considers three different attributions of people: college students [17], pregnant women [18], and hospital nurses [19], using the Japanese version of the FCV-19S and the risk-factor item [16].

During the pandemic, college students experienced many disruptions and social changes. Many college students were forced to study at home and experienced reduced social interaction due to COVID-19 [20]. In Japan, many university lectures are online, and college students have reported experiencing anxiety in all aspects of their lives, including self-restraint, university life, financial activities, club activities, and the future [21]. As a result, worsening mental health among college students has been reported in many countries, with a meta-analysis showing that 29% of college students have depressive symptoms and 23% have stress symptoms [22]. In addition, many studies have found that COVID-19-related anxiety includes a moderate fear of infection [23–25]. Under these social conditions, a Japanese study [17] surveyed college students using items developed by Wakashima et al. [16], it examined the relationship between family members, information sources, psychological and social behaviors, and fear of infection. The results showed that fear of infection was associated with psychological and social behaviors, including avoidance of interpersonal contact, stockpiling, and health monitoring, among college students.

By contrast, older people and pregnant women are referred to as “high-risk individuals,” who are especially vulnerable to the virus [26]. Pregnant women, in particular, not only have a high likelihood of becoming severely ill when infected with COVID-19, but are also at risk for preterm birth [27]. Moreover, pregnant women have been found to experience more serious mental health problems during the pandemic, given their vulnerability [28]. Studies in Iran showed that fear of infection in pregnant women decreases the quality of life [29], worsens mental health [30], and increases depressive symptoms and suicide attempts [31]. A study of pregnant women in Japan [18] surveyed pregnant women, using items developed by Wakashima et al. [16] to investigate the relationship between family members, information sources, psychological and social behaviors, and fear of infection. The results showed that non-traditional media, including social networking sites (SNS), could alleviate the fear of infection more effectively than traditional media, such as newspapers and TV.

Healthcare workers, including hospital nurses, are believed to have a significant fear of infection [32] because they have a high risk of coming into contact with infected persons; healthcare workers account for approximately 10% of COVID-19 cases worldwide [33]. Among Iranian hospital nurses, 30.4% reported mild to moderate anxiety, and 21.3% had severe anxiety symptoms [34]. Other reports from Taiwan indicated that 15% of healthcare workers developed post-traumatic stress disorder, 25.6% depression, 23.4% stress reactions, and 30.6% anxiety symptoms [35]. In a meta-analysis of healthcare workers’ mental health during the COVID-19 pandemic, the prevalence of sleep disorders was 43% [4]. Serious mental health problems have been reported among healthcare workers.

Among healthcare workers, hospital nurses have been at the forefront of medical care during the pandemic, playing a central role [36]. Fear of infection is the most significant stressor faced by hospital nurses working in harsh conditions [37], leading to sleep disturbances, psychological distress, decreased job satisfaction, and turnover intention among hospital nurses [38, 39]. In this social context, a study of hospital nurses in Japan [19] has surveyed hospital nurses, using items developed by Wakashima et al. [16] to explore the relationship between family members, information sources, psychological and social behaviors, and the fear of infection. The results show that hospital nurses who live with older people have a particularly high fear of infection [19].

As discussed above, research on fear of infection in Japan have evolved to include people in different attributions: college students who have experienced social disruption [17], pregnant women at high risk [18], and hospital nurses, who are healthcare workers [19]. However, these studies leave several issues unanswered. First, they do not compare the fear of infection among different attributions. Although two studies have measured the fear of infection by comparing participant scores with those of subjects in foreign countries [17, 19], it is important to compare differences in the fear of infection among groups of people in the same country, using statistical methods. Second, since it is unclear whether the fear of infection and its determinants are unique to each attribution, such data must also be compared with general-population data. The third issue involves the unification of statistical methods and the treatment of variables. For example, Asai et al. [18] grouped major information sources into “traditional media” and “non-traditional media” before analyzing them. In other studies [17, 19], there was no such manipulation. Since the analytical method and variables are handled differently from study to study, a unified method of analysis is needed.

The purpose of this study is therefore to compare the fear of infection and related factors among different attributions of Japanese people from various social standpoints. First, we surveyed Japanese people, excluding college students, pregnant women, and hospital nurses; this group was referred to as “the general public.” We also used data from previous studies dealing with college students [17], pregnant women [18] and hospital nurses [19]. Based on this, we examined the fear of infection and related factors among college students, pregnant women, and hospital nurses, and using the general public as the baseline.

## Method

### Survey participants

An online survey was carried out to establish fear-of-infection levels in the general public, and 450 responses were obtained. For comparison, we used data from a previous FCV-19S-based study conducted in Japan at the same time. Three studies, Takagi et al. [17], Asai et al. [18], and Koiwa et al. [19] were conducted using web-based surveys about fear of COVID-19. For hospital nurses (N = 152), pregnant women (N = 318), and college students (N = 300), were selected from these data. As a result, 1220 data were obtained in this way.

### Fear of infection among members of the general public

#### Procedure

The data were collected within Japan. The participants were 450 Japanese residents (286 men and 164 women) aged 18 or above, with a mean age of 48.34 years (SD = 14.07). The participants were recruited using a major crowdsourcing service in Japan, operated by Yahoo Japan Corporation (https://crowdsourcing.yahoo.co.jp/). This service connects client requests with crowdsourced workers. The authors posted the present study on the Yahoo Information Bulletin Board in the “Questionnaire” category, describing it as a psychology research project. The number of survey participants was capped when 450 participants had signed up. The participants read a description of the study and agreed to participate by opting themselves in. Those who completed the survey received 105 points (approximately $1.00) to use at selected stores. The survey period ran from June 8 to June 9, 2020.

### The fear of COVID-19 Scale (FCV-19S)

The FCV-19S, developed by Wakashima et al. [16] was used to assess the fear of COVID-19. Participants responded to items using a five-point Likert-type scale, with responses ranging from 1 (strongly disagree) to 5 (strongly agree). Totaling the individual response items created total sums between 7 and 35, with higher scores indicating a more pronounced fear of COVID-19 [16].

#### Psychological and social behavior

The respondents were asked about their COVID-19-related behavior. A previous study [16] developed 19 items for measuring COVID-19-coping behavior, based on a report from the Ministry of Health, Labor and Welfare [40] and a newspaper article on social issues [41]. The present study used the 19 items [16] as a scale of COVID-19-related behavior. Each item was rated using a 6-point scale, with responses ranging from 1 (not at all) to 6 (very much). The items were analyzed by Wakashima et al. [16] and grouped into three categories: “being careful in daily life” (continuing preventive actions against COVID-19), “stockpiling” (buying and stockpiling food and daily necessities), and “health monitoring” (observing one’s own health status).

#### Demographic variables and risk factors

In addition to FCV-19S, the present study investigated demographic variables and risk factors related to fear of infection, as described by Wakashima et al. [16]. The demographic variables included age, smoking history, and family structure. The risk factors included items related to current health status, any illness being treated, employment status, family communication during the last month, family conflict during the last month, key sources of information, the presence of infected people in your area (prefecture), the presence of infected acquaintances, and motivations of choosing COVID-19-related coping behaviors and motivations. Overall, 11 healthcare workers, 4 students, and 1 pregnant woman were excluded from the analysis; the remaining 434 (282 men and 152 women, with a mean age of 48.72 years, SD = 13.91) were included in the analysis.

#### Ethical considerations

Written informed consent was obtained before the investigation was initiated. Specific tasks included the following. The following information was included on the survey cover page. The participants were informed of the purpose of the survey. They were told that participation was voluntary, that the survey was anonymous, and that personal information would not be disclosed to third parties. After explaining this information in writing, the respondents were given the option of “agreeing to participate in the survey” or “not agreeing to participate in the survey” in their responses to the questionnaire. The questionnaire was set up such that those who chose the latter option would complete the survey as it is, thereby confirming that informed consent was obtained. Additionally, minors were not included in the survey.

### Fear of infection among college students

For the college-student data, we used the dataset from Takagi et al. [17]. This survey included college students from all over Japan, considering family factors, key sources of information, items related to psychological and social behavior, and FCV-19S. The participants were 52 men and 248 women (mean age: 19.80, SD = 1.36). After confirming that no participants were pregnant and excluding incomplete responses, the data of all participants were used in the analysis. The study period ran from May 10 to June 14, 2020.

### Fear of infection among pregnant women

For the pregnant women’s data, we used the Asai et al. [18] dataset. This survey included pregnant women from all over Japan, considering family factors, key sources of information, items related to psychological and social behavior, and FCV-19S. A total of 404 pregnant women living in Japan were included in the study. Of these, 292 pregnant women (mean age 31.18, SD = 3.85) were included in the analysis, after 112 women with description errors were excluded. The study period ran from May 21, 2020 to May 31, 2020.

### Fear of infection among hospital nurses

The Koiwa et al. [19] dataset was used for the hospital nurses’ data. That study surveyed 152 hospital nurses (mean age 37.47 years, SD = 11.61, 1 age non-response, 9 men and 142 women) working in a hospital in the Tohoku region of Japan. The survey included items on family factors, key sources of information, and psychosocial behavior. Of these, eight participants with errors and two who were pregnant were excluded; the remaining 142 participants (mean age 37.75, SD = 11.57, 9 men, 133 women) were included in the analysis. The study period ran from May 20, 2020 to June 5, 2020. The basic demographics of the general public, college students, pregnant women, and hospital nurses included in the analysis, respectively, are shown in Table 1.

**Table 1:** Respondent demographics.

	General Public(N = 434)	College Student (N = 300)	Pregnant Woman (N = 292)	Hospital Nurse(N = 142)
**Age**				
−29	34	300	107	51
30≤	108	0	178	27
40≤	97	0	7	37
50≤	51	0	0	25
60≤	119	0	0	1
70≤	25	0	0	0
**Gender**				
Men	282	52	0	9
Women	152	248	292	133
**Employment Status**				
Full-time worker	216	――	182	138
Part-time worker	66		21	4
Unemployed	152		42	0

Employment Status of college students has been omitted because all respondents were unemployed. Employment Status among pregnant women includes 47 persons on Maternity Leave in addition to the "Full-time," "Part-time," and "Unemployed" categories listed in the table.

#### Infection situation in Japan

All of the surveys in this study were carried out between May 10 and June 14. The infection status in Japan during this period can be deduced from Ministry of Health, Labor and Welfare data [2]. In Japan, a domestic case was confirmed on January 29, 2020, and the number of infected people continued to increase until April. In response, the Japanese government declared a state of emergency in seven major prefectures on April 7, 2020, and expanded the scope of the emergency to the entire country on April 16, 2020. However, the number of new infections began to decrease on April 11. The average number of newly infected persons per day during the survey period was 44.6 (minimum 22, maximum 99), while the nationwide declaration of a state of emergency was lifted on May 25, during the survey period. In light of the above, it can be said that the first wave of the pandemic had begun to subside in Japan at the time of the survey.

#### Data analysis

All analyses were conducted using IBM SPSS statistical-analysis software (version 25). In every statistical evaluation, a p-value of less than 0.05 was thought to indicate a significant difference.

The following is a description of how the variables of the relevant factors are handled. First, among information sources, newspapers and TV news/talk shows were categorized as the traditional-media viewing group, while public websites, Internet news, and social networking sites were categorized as the Internet/social-media use group, based on Asai et al. [18]. The traditional-media viewing group was assigned a value of “0,” while the Internet/social-media use group was assigned a value of “1.” When considering the risk to older people, respondents who lived with a family member aged 65 or above were assigned a value of “1,” while those who did not were assigned a value of “0.” Both Wakashima et al. [16] and Takagi et al. [17] treated psychosocial behavior as a dependent variable, while Asai et al. [18] and Koiwa et al. [19] treated psychosocial behavior as an independent variable. The present study has adopted the latter approach, treating psychosocial behavior as an explanatory variable in the multiple regression analysis.

## Results

### A comparison of levels of fear of infection

To compare the level of fear of infection by attribution, a one-factor between-subjects analysis of variance was conducted using each attribute (hospital nurse, college student, the general public, pregnant woman) as the independent variable and the fear of infection score as the dependent variable (see Table 2). There was thus a difference in fear of infection by attribution (F (3, 1164) = 54.59, p < .001, F068p^2^ = .12). Multiple comparisons using the Turkey method showed no significant difference between the general public and hospital nurses. By contrast, in comparison to members of the general public, college students had less fear of infection (p < .01), while pregnant women had more fear of infection (p < .001). There were also significant differences between college students and pregnant women and between hospital nurses and pregnant women (p < .001).

**Table 2:** Comparing the fear of infection by attribution.

	General public (N = 434)	College student (N = 300)	Pregnant woman (N = 292)	Hospital nurse (N = 142)	F
M	19.00	17.88	22.96	18.27	54. 59***
SD	5.28	4.95	5.68	5.13	

*** p < .001

### Comparison of factors associated with the fear of infection

A multiple regression analysis was conducted to clarify the relationship between each variable and the fear of infection. Only variables that were found to be significantly related in previous studies [16–19] were used in the multiple regression analysis. The following five variables were used as explanatory variables: (a) key sources of information, (b) the presence of older people at home, (c)“being careful in daily life,” (d) “stockpiling,” and (e) “health monitoring.”

A multiple regression analysis, based on the forced-entry method, was conducted for each attribution, with five explanatory variables and the fear of infection as the objective variable (see Table 3). In both analyses, the VIF values for each explanatory variable ranged from 1.01 to 1.45, indicating that multicollinearity was unlikely to be indicated. The results were as follows: First, among members of the general public, there was a positive association (R^2^ = .20, p < .001) with “health monitoring” (β = .36, p < .001, 95%CI [.42, .74]). Second, among college students, the key source of information (β = -.13, p < .05, 95%CI [-.24, -.18]) was negatively associated with fear (R^2^ = .04, p < .01). Among pregnant women, the key source of information (β = -.12, p < .05, 95%CI [-.26, -.21]) was negatively associated with fear, while “stockpiling” (β = .11, p < .05, 95%CI [.01, .48]) and “health monitoring” (β = .38, p < .01, 95%CI [.57, 1.06]) were positively associated with fear (R^2^ = .22, p < .001). Finally, among nurses, there was a positive association between living with an older family member (β = .19, p < .05, 95CI [.33, 4.92], "health monitoring" (β = .19, p < .05, 95%CI [.05, .72]), and fear (R^2^ = .14, p < .001).

**Table 3:** Related factors of fear of infection for each attribution.

	The general public (N = 434)	College student (N = 300)	Pregnant woman (N = 292)	Hospital nurse (N = 142)
Key sources of information (Traditional 0, non-traditional 1)	-.00	-.13*	-.12*	-.15
Older family members living with participant (No 0, Yes 1)	.00	-.02	-.08	.19*
“Careful in daily life”	.09	.07	.06	.12
"Stockpiling"	.09	.02	.11*	.14
“Health monitoring”	.36***	.09	.38***	.19*
R^2^	.20***	.04**	.22***	.14***

* p < .05,

** p < .01,

*** p < .001

## Discussion

The present study has focused on the fear of infection among Japanese people, comparing the fear of infection among people in different attributions: members of the general public, college students, pregnant women, and hospital nurses. The results show that pregnant women have more fear of infection than members of the general public and college students, in that order, while hospital nurses have the same level of fear as members of the general public. Based on descriptive statistics, previous studies have shown that college students have a moderate fear of infection [23–25]. By contrast, the present study, which has controlled for timing factors and compared results within Japan, reveals that the fear of infection is relatively low among college students. This result may reflect the limited social interactions among college students. In Japan, many university lectures were online and many students were required to stay at home during the pandemic. For this reason, at the time of the survey, college students had few social interactions [20, 21]. In addition, COVID-19 is more likely to make older people severely ill, while the levels of severity are relatively low in the younger age group [26]. As described above, given a relatively low risk of contact with infected people and serious illness if infected, Japanese college students had a relatively low fear of infection.

Second, pregnant women were found to have a more pronounced fear of infection than members of the general public, college students, or hospital nurses. According to Asai et al. [18] pregnant women in Japan were more fearful of infection than pregnant women in other countries; in the present study, they were more fearful of infection than other Japanese. This result may reflect the characteristics of COVID-19, which causes a high incidence of severe disease in pregnant women, with the associated risk of miscarriage [27]. In other words, high-risk individuals, including pregnant women, are particularly vulnerable to natural disasters and large-scale disease epidemics [43] and thus have a more pronounced fear of infection.

By contrast, among hospital nurses, the fear of infection was lower than that of pregnant women; in fact, it did not differ significantly from that of the general public and college students. Hospital nurses are at a higher risk of coming into contact with patients infected with COVID-19 [33]; previous studies have found that health care worker have a particular fear of infection [5]. The present results were not consistent with those findings. Contrary to these findings, a study comparing the fear of infection between the general public in Hong Kong and healthcare workers in Taiwan revealed that the former was more fearful [42]. Furthermore, Alimoradi et al. [4] asserted that the incidence of sleep disturbances in male healthcare workers is not different from that in the general population. These are signs that the public perception of nurses’ mental health and fear of infection may be overstated, in some countries and regions. There are three possible explanations for this discrepancy. The first involves the timing of the survey, which was carried out at a time when the level of infection was temporarily stable [2]. For this reason, the hospital nurses may have been less afraid of catching COVID-19. Second, they may have been emotionally numb. Previous studies of infectious diseases have found that exposure to a large amount of infection-related information can lead to emotional numbing and reduced fear [44]. The workplace of the hospital nurses was flooded with information about COVID-19 during the pandemic; this may have caused emotional numbing and prevented them from fearing infection. The third explanation involves appropriate coping strategies. Hospital nurses are expected to have more specialized skills and knowledge of COVID-19 prevention and treatment than other people. We can speculate that this appropriate knowledge and methods of dealing with COVID-19 may have contributed to the low fear of infection among hospital nurses.

The present study also compared factors associated with the fear of infection. First, the association between psychosocial behaviors among members of the general public and the fear of infection was significant for “health monitoring,” but not for “being careful in daily life” or “stockpiling.” These results were similar for the hospital nurses. Compared to Wakashima et al. [16], which was conducted during the early stages of the pandemic, the data used in this study were collected during a lull in the spread of infection [2]. It can therefore be inferred that participants temporarily avoided selecting “being careful in daily life” and “stockpiling.”

In addition, pregnant women showed an association between "health monitoring" among psychosocial behaviors and fear of infection. While studies of pregnant women in Iran have shown an association between fear of infection and preventive behaviors [31], this study was consistent in that fear and "health monitoring" were significantly associated. While Ahorsu et al. [31] noted that Iranian pregnant women had correctly implemented procedures to protect themselves from COVID-19, it was suggested that Japanese pregnant women were also attempting to do so by properly managing their health. Moreover, only the pregnant women showed an association between “stockpiling” and fear of infection. They refrained from going out because of their significant fear of infection and tended to buy many necessary items at once. By contrast, the fear of infection was not associated with any of these behaviors among college students; as COVID-19 is thought to be less severe in younger people [26], their fear of infection was lower and did not lead to infection prevention behaviors.

As for the association between other risk factors and the fear of infection, living with an older family member was a significant factor for hospital nurses, but not for members of the general public. This finding suggests that such results are characteristic of hospital nurses. The finding that nurses living with older adults have a higher fear of infection is consistent with that of Tercan et al. [37], that living with high-risk individuals is a factor in nurses’ anxiety. The reason for this is believed to be that hospital nurses worry about being a source of infection and spread it to others [32, 45]. In addition, older people are at high risk of becoming seriously ill if infected [26], and hospital nurses who live with them may be especially fearful. For this reason, hospital nurses with older family members are especially afraid of becoming a source of infection themselves, and thus have a high fear of infection.

Moreover, the association between critical sources of information and fear of infection was only significant among pregnant women and college students. This study showed no association with anything other than information resources and was consistent with the finding that information resources were the sole predictor of anxiety among Taiwanese college students [46]. Conversely, in previous studies, social mediation has been considered a factor that worsens mental health [47]. The acquisition of internet information may lead to a low fear of infection, which may be a phenomenon unique to Japan. Hasannia et al. [34] reported cultural differences in information circulated on the Internet. Accordingly, we speculate that there may have been information on social networking sites in Japan, suggesting that COVID-19 was not to be feared.

Although it has been pointed out that traditional media such as newspapers and television may increase fear among pregnant women [18], the same result was observed among college students. It can thus be inferred that pregnant women and college students share the condition of little interpersonal contact. For this reason, they may be more likely to receive informational influence from traditional media, which may arouse fear of infection.

### Limitations

This study has several limitations. The first involves the timing of the study, which ran from May to June 2020; in Japan, the spread of infection temporarily decreased during this period [2]. The timing of the survey must be considered because the fear of infection among hospital nurses was expected to be higher during this medical emergency. Second, the control of these factors is important. In this study, cultural and timing-related factors were controlled to allow the fear of infection to be compared by attribution. However, the present study did not control for basic factors, such as age, gender, or region. Future studies should consider the effects of these factors.

## Conclusion

The present study set out to compare the fear of infection among different attributions of Japanese people. We compared fear of infection and related factors among members of the general public, college students, pregnant women, and hospital nurses. The results showed that fear of infection was higher among pregnant women, lower among college students, and equivalent among hospital nurses and members of general public. It was also revealed that college students and pregnant women associated the fear of infection with their key source of information, while hospital nurses associated the fear of infection with living with an older person. The fear of infection with COVID-19 is an important problem in modern society. Understanding which people, factors, and levels of fear of infection are most significant will help to provide psychological support to key groups.

## Supporting information

S1 Dataset (XLSX)
